# Shared Molecular Mechanisms between Atherosclerosis and Periodontitis by Analyzing the Transcriptomic Alterations of Peripheral Blood Monocytes

**DOI:** 10.1155/2021/1498431

**Published:** 2021-12-03

**Authors:** Wanchen Ning, Yihong Ma, Simin Li, Xin Wang, Hongying Pan, Chenxuan Wei, Shaochuan Zhang, Dongying Bai, Xiangqiong Liu, Yupei Deng, Aneesha Acharya, George Pelekos, Vuk Savkovic, Hanluo Li, Sebastian Gaus, Rainer Haak, Gerhard Schmalz, Dirk Ziebolz, Yanbo Ma, Yuzhen Xu

**Affiliations:** ^1^Stomatological Hospital, Southern Medical University, Guangzhou 510280, China; ^2^Department of Neurology, Graduate School of Medical Sciences, Faculty of Life Sciences, Kumamoto University, Kumamoto, Japan; ^3^Department of Neurology, First Affiliated Hospital of Harbin Medical University, Harbin 150001, China; ^4^School of Dentistry, University of Michigan, 1011 N University Ave, Ann Arbor, MI 48109, USA; ^5^Division of Neurogenetics, Center for Neurological Diseases and Cancer, Nagoya University Graduate School of Medicine, Nagoya, Japan; ^6^College of Animal Science and Technology, Henan University of Science and Technology, Luoyang 471003, China; ^7^Laboratory of Molecular Cell Biology, Beijing Tibetan Hospital, China Tibetology Research Center, 218 Anwaixiaoguanbeili Street, Chaoyang, Beijing 100029, China; ^8^Dr D Y Patil Dental College and Hospital, Dr D Y Patil Vidyapeeth, Pimpri, Pune, India; ^9^Faculty of Dentistry, University of Hong Kong, Hong KongChina; ^10^Department of Cranio Maxillofacial Surgery, University Clinic Leipzig, Liebigstr. 12, 04103 Leipzig, Germany; ^11^Department of Cariology, Endodontology and Periodontology, University of Leipzig, 04103 Leipzig, Germany; ^12^Department of Rehabilitation, The Second Affiliated Hospital of Shandong First Medical University, Taian, Shandong Province 271000, China

## Abstract

**Objective:**

This study investigated the nature of shared transcriptomic alterations in PBMs from periodontitis and atherosclerosis to unravel molecular mechanisms underpinning their association.

**Methods:**

Gene expression data from PBMs from patients with periodontitis and those with atherosclerosis were each downloaded from the GEO database. Differentially expressed genes (DEGs) in periodontitis and atherosclerosis were identified through differential gene expression analysis. The disease-related known genes related to periodontitis and atherosclerosis each were downloaded from the DisGeNET database. A Venn diagram was constructed to identify crosstalk genes from four categories: DEGs expressed in periodontitis, periodontitis-related known genes, DEGs expressed in atherosclerosis, and atherosclerosis-related known genes. A weighted gene coexpression network analysis (WGCNA) was performed to identify significant coexpression modules, and then, coexpressed gene interaction networks belonging to each significant module were constructed to identify the core crosstalk genes.

**Results:**

Functional enrichment analysis of significant modules obtained by WGCNA analysis showed that several pathways might play the critical crosstalk role in linking both diseases, including bacterial invasion of epithelial cells, platelet activation, and Mitogen-Activated Protein Kinases (MAPK) signaling. By constructing the gene interaction network of significant modules, the core crosstalk genes in each module were identified and included: for GSE23746 dataset, RASGRP2 in the blue module and VAMP7 and SNX3 in the green module, as well as HMGB1 and SUMO1 in the turquoise module were identified; for GSE61490 dataset, SEC61G, PSMB2, SELPLG, and FIBP in the turquoise module were identified.

**Conclusion:**

Exploration of available transcriptomic datasets revealed core crosstalk genes (RASGRP2, VAMP7, SNX3, HMGB1, SUMO1, SEC61G, PSMB2, SELPLG, and FIBP) and significant pathways (bacterial invasion of epithelial cells, platelet activation, and MAPK signaling) as top candidate molecular linkage mechanisms between atherosclerosis and periodontitis.

## 1. Introduction

Much epidemiological evidence has highlighted the causal relationship between periodontitis and atherosclerosis, suggesting periodontitis an independent risk factor that contributes to the development of atherosclerosis [1]. This causal linkage between the two diseases has been attributed to two major mechanisms: a direct mechanism, whereby periodontal pathogens invade the vessel walls, and an indirect mechanism of systemic inflammatory responses that are triggered by periodontitis leading to inflammatory mediator enhancement [2]. These inflammatory mediators include C-Reactive Protein (CRP), interleukin- (IL-) 6, IL-8, cytokines and chemokines, Matrix Metalloproteinases (MMPs), reactive oxygen species (ROS), nitric oxide, and thrombotic and hemostatic markers (fibrinogen) [1].

Systemic inflammation constitutes a major linkage between periodontitis and atherosclerosis, albeit both diseases also share several common risk factors such as aging, smoking, alcohol abuse, race/ethnicity, educational and socioeconomic status, male sex, diabetes mellitus, overweight/obesity, and genetic susceptibility [3]. Common genetic risk factors in periodontitis and atherosclerosis that may predispose certain individuals to suffer both diseases have been identified [4, 5]. A twin study from Sweden using quantitative genetic analyses identified significant genetic correlation between periodontitis and atherosclerosis [4]. Others, using genome-wide association (GWAS) identified three genetic variants CDKN2B Antisense RNA 1 (CDKN2B-AS1), Plasminogen (PLG), and Vesicle- Associated Membrane Protein 3 (VAMP3) as significant to both diseases [5]. However, a broader understanding of shared genetic and molecular links between these diseases is largely lacking. To the authors' knowledge, comprehensive and integrated bioinformatic analyses of disease-related datasets in Gene Expression Omnibus (GEO) database [6] and disease-related known genes in the DisGeNET database [7] to unravel potentially shared molecular mechanisms in this context have not been reported.

Peripheral blood monocytes (PBMs), as innate immune effector cells, play critical roles in the initiation and development of both periodontitis and atherosclerosis. In periodontitis, phenotypical alterations of PBMs compared to those from periodontal healthy subjects are recognized, showing a specific functional profile favoring T-helper- (Th-) 2 cell response over Th-1 cell response [8]. Using RNA-seq data (GSE41690), transcriptomic alterations in PBMs from periodontitis patients were compared with PBMs of periodontal healthy subjects [9]. In case of atherosclerosis, PBMs are reported to be in an activated state and respond more strongly against lipopolysaccharide (LPS) stimulation, showing the increased expression of inflammatory mediators [10]. A publicly available microarray dataset (GSE23746) pertains to transcriptomic aberrations occurring in the PBMs of atherosclerosis patients versus the systemically healthy subjects. Regarding periodontitis-associated atherosclerosis, a previous animal study found that ligature-induced periodontitis could activate PBMs and result in significant upregulation of proinflammatory genes including Tumor Necrosis Factor Alpha (TNFɑ) and IL-6 in PBMs to increase the adhesion of PBMs to the aortic endothelium, finally triggering the initiation of atherosclerosis [11]. These findings suggest that PBMs might serve as key linkage cells between periodontitis and atherosclerosis. Thus, this study put forwarded to a hypothesis that the transcriptomic alterations in PBMs seen in periodontitis and atherosclerosis may have shared features.

In order to validate this hypothesis, the current study is aimed at investigating gene expression profiling data from periodontitis- and atherosclerosis-linked datasets, identifying the periodontitis- and atherosclerosis-related known genes in the DisGeNET database, and performing a series of comprehensive bioinformatics analyses to reveal key genes, biological processes, and signaling pathways that could be regarded as molecular links between periodontitis and atherosclerosis. Such data can enable improved understanding of the pathophysiological links between the two diseases and uncover valuable targets for risk assessment or drug development in this context.

## 2. Methods

### 2.1. Data Procurement

Gene expression datasets investigating the PBMs of periodontitis (GSE61490) and atherosclerosis (GSE23746) were each sourced and downloaded from the NCBI GEO [6]. GSE61490 investigated gene expression patterns of PBMs in patients with periodontitis versus periodontal healthy controls (URL: https://www.ncbi.nlm. http://nih.gov/geo/query/acc.cgi?acc=GSE61490). GSE23746 investigated altered gene expression of PBMs among patients with atherosclerosis compared to healthy controls (URL: https://www.ncbi.nlm.nih.gov/geo/query/acc.cgi?acc=GSE23746). The diagnosis of periodontitis should be defined in accordance with the case definitions for periodontitis in the context of the 2017 world workshop on the classification of periodontal disease: interdental CAL detectable at ≥2 nonadjacent teeth or buccal or oral CAL ≥ 3 mm with pocketing > 3 mm detectable at ≥2 teeth [12].

### 2.2. Differential Expression Analysis

Differential expression analysis was performed for the GSE23746 dataset using the bioconductor package “limma” in R program [13, 14]. The specified cutoff criteria for differentially expressed genes (DEGs) were *p* value < 0.05 and ∣log FC | ≥0. RNA seq data from GSE61490 was mapped to the human genome using TopHat [15]. Qualification of the mapped reads and the differential expression analysis were conducted using Cufflinks [14], where genes with a *p* value < 0.05 and ∣log FC | ≥0.5 were selected as DEGs. By overlapping the DEGs dysregulated in the atherosclerosis-GSE23746 and DEGs dysregulated in the periodontitis-GSE61490 dataset, the Venn diagram was plotted using a specialized web tool (URL: http://bioinformatics.psb.ugent.be/webtools/Venn/). These overlapped DEGs were dysregulated in both GSE23746 and GSE61490 dataset and thus were defined as candidate crosstalk genes linking atherosclerosis and periodontitis.

### 2.3. Functional Enrichment Analysis

The functional enrichment analyses were carried out in order to investigate the Gene Ontology (GO) terms, particularly biological processes (BPs), and Kyoto Encyclopedia of Genes and Genomes (KEGG) pathways enriched by the candidate crosstalk genes-overlapping DEGs. This analysis was performed with the “ClusterProfiler” package in R program [16]. The functional terms with statistical significance *p* value< 0.05 were selected as significant functions. The top 30 enriched BPs and KEEG pathways were visualized in bar plots.

### 2.4. Construction of Protein-Protein Interaction (PPI) Network

The PPI network was constructed using the candidate crosstalk genes-overlapping DEGs dysregulated in both the atherosclerosis-GSE23746 and periodontitis-GSE61490 datasets. Experimentally validated PPI pairs were downloaded from several databases including HPRD [17], BIOGRID [18], DIP [19], MINT [20], mentha [21], PINA [22], InnateDB [23], and Instruct [24]. The PPI network was then constructed with the “Cytoscape” software [25], and the topological features were analyzed using the “NetworkAnalyzer” plugin in Cytoscape to identify hub genes. The top 30 nodes were selected based on descending order of degree.

### 2.5. Identification of Crosstalk Genes by Integrating GEO Datasets and Disease-Related Known Genes in DisGeNET Database

The periodontitis-related and atherosclerosis-related known genes were, respectively, obtained from the DisGeNET database (version 6.0) [26]. By now, four groups of genes were collected:

*Group A*: DEGs dysregulated in the atherosclerosis-GSE23746 dataset

*Group B*: DEGs dysregulated in the periodontitis-GSE61490 dataset

*Group C*: the periodontitis-related known genes (UMLS CUI: C0031099) obtained from DisGeNET database

*Group D*: the atherosclerosis-related known genes (UMLS CUI: C0004153) obtained from the DisGeNET database

In order to visualize the overlap between these four sets of genes, a Venn diagram was plotted with the above mentioned web tool.

The crosstalk genes were generated from this Venn diagram by the following two steps: Firstly, the intersections of gene group belonging to periodontitis and gene group belonging to atherosclerosis were obtained: for example, intersection between group A and group B (A∩B), intersection between group C and group D (C∩D), intersection between group A and group C (A∩C), and intersection between group B and group D (B∩D). It is important to emphasize that the intersection between two gene groups belonging the same disease will not be regarded as crosstalk genes, which means the intersection between group A and group D (A∩D) and intersection between group B and group C (B ∩ D) will be included. Secondly, all these intersection genes (A∩B, C∩D, A∩C, and B∩D) were taken together as a union, the genes of which was regarded as the crosstalk genes.

Afterward, the expression profile of periodontitis-related known genes in the atherosclerosis-GSE23746 dataset, as well as the expression profile of atherosclerosis-related known genes in the periodontitis-GSE61490 dataset was extracted and displayed using the pheatmap package in R program [27].

### 2.6. Identification of Coexpression Modules

The weighted correlation network analysis (WGCNA) was constructed for the genes in the atherosclerosis-GSE23746 dataset (adj.P.Val (*p* value)<0.05) and periodontitis-GSE61490 dataset (*p* value < 0.05), respectively. The “wgcna” package in R was applied to construct the coexpression network and further to identify the coexpression gene modules, according to previously described methodology for WGCNA analysis [28]. Briefly, an unsupervised coexpression relationship was initially built based on the adjacency matrix of connection strengths using Pearson's correlation coefficients for gene pairs. Then, the power *β* was calculated, using the “pickSoftThreshold” function. Based on the scale-free topology criterion, the optimum power *β* was selected to amplify the strong connections between genes and penalize the weaker connections. In addition, the hybrid dynamic tree cutting method was used to cut branches and cluster coexpression modules in the GSE23746 (cutHeight = 0.97, minSize = 20) and GSE61490 (cutHeight = 0.9, minSize = 20).

### 2.7. Identification of Significant Modules

The crosstalk genes of the above described coexpression modules were extracted and overlapped between any one coexpression module in the atherosclerosis-GSE23746 and peridoontitis-GSE61490. The Fisher's exact probability test was used to validate the significance of the overlapping across coexpression modules, and a heat map was plotted. The significant modules met the following two criteria: first, the Fisher_p value between two modules was less than 0.001, and grey unassigned module was not considered; second, the proportion was more than 50% in at least either one module.

### 2.8. Biological Functions of Crosstalk Genes in the Significant Modules

The expression profiles of the crosstalk genes identified in the different significant modules were obtained and depicted using the “pheatmap” package in R. Next, functional enrichment analysis was performed to identify the significant BPs and KEGG pathways enriched by the above crosstalk genes using the “clusterProfiler” package in R [16].

### 2.9. Identification of the Core Crosstalk Genes

The final step was aimed at identifying the core crosstalk genes. In order to achieve this objective, the genetic interactions among the crosstalk genes were investigated for the different significant modules. The top 50 crosstalk genes were selected for each module, based on the descending order of the intramodular connectivity values. If there were less than 50 crosstalk genes in a certain module, then all crosstalk genes were used as the input. If there were more than 50 crosstalk genes in a certain module, then top 50 crosstalk genes were taken as the input. Next, coexpression networks for each significant module were visualized with the “Cytoscape” software [25], based on the all interaction pairs consisting of the crosstalk genes. The crosstalk genes that were dysregulated in both periodontitis-GSE61490 dataset and atherosclerosis-GSE23746 dataset were regarded as the core crosstalk genes.

## 3. Results

### 3.1. The Study Design of the Present Research

As shown in Figure 1, the present study included four major steps. Step 1 was aimed at identifying the candidate crosstalk genes by overlapping the DEGs dysregulated in both the periodontitis-GSE61490 dataset and atherosclerosis-GSE23746 dataset. Step 2 was aimed at identifying the crosstalk genes by taking together all intersecting genes between pairs of four gene sets: DEGs dysregulated in periodontitis-GSE61490 dataset, DEGs dysregulated in the atherosclerosis-GSE23746 dataset, periodontitis-related known genes in DisGeNET database, and atherosclerosis-related known genes in DisGeNET database. In the step 3, a WGCNA analysis was performed to identify coexpression modules in the GSE61490 dataset and GSE23746 dataset; of these, four significant coexpression modules with high correlation were identified. In step 4, by extracting the expression profile of the crosstalk genes (obtained in the step 2) in the significant modules, the crosstalk gene interaction networks were constructed for the four different significant modules.

### 3.2. 165 DEGs That Were Dysregulated in Both Periodontitis and Atherosclerosis

By performing differential expression analysis, a total of 1,170 DEGs consisting of 382 upregulated DEGs and 788 downregulated DEGs were identified to be involved in periodontitis, while a total of 2,621 DEGs consisting of 1,413 upregulated DEGs and 1,208 downregulated DEGs were identified as involved in atherosclerosis. As shown in the Venn diagram (Figure 2(a)), 165 DEGs were found to be dysregulated in both periodontitis and atherosclerosis, by overlapping the DEGs identified in periodontitis-GSE46190 dataset and atherosclerosis-GSE23746 dataset.

### 3.3. PPI Network of the 165 Overlapping DEGs

Based on the 165 DEGs overlapping between periodontitis-GSE46190 dataset and atherosclerosis-GSE23746 dataset, a PPI network shown in Figure 2(b) was constructed and was consisted of 6,212 nodes and 11,202 edges. The topological characteristics of the top 30 nodes ranked in the descending order of degree are displayed in Table 1. The purple nodes in Figure 2(b) represent the DEGs dysregulated in both GSE46190 and GSE23746 datasets. Among these, the purple nodes with the greatest degrees were found to be the gene Amyloid Beta Precursor Protein (APP), Small Ubiquitin Like Modifier 1 (SUMO1), GABA Type A Receptor Associated Protein Like 1 (GABARAPL1), SRC Proto-Oncogene, Nonreceptor Tyrosine Kinase (SRC), Casein Kinase 2 Beta (CSNK2B), and OFD1 Centriole And Centriolar Satellite Protein (OFD1) (Table 1). These genes interacted with the greatest number of other DEGs in the PPI network, thus might play critical roles in the crosstalk between both diseases.

### 3.4. Biological Processes and Signaling Pathways Enriched by the 165 Overlapping DEGs

The 165 overlapping DEGs shared between periodontitis-GSE46190 dataset and atherosclerosis-GSE23746 dataset were significantly enriched in several biological processes, for example, cellular response to hydrogen peroxide and increased oxygen levels, neutrophil activation and degranulation, regulation of leukocyte activation, platelet degranulation, positive regulation of chemokine biosynthetic process, and cellular response to antibiotic (Figure 2(c)). In addition, these overlapping DEGs were also significantly enriched in multiple signaling pathways, including spliceosome, platelet activation, bacterial invasion of epithelial cells, human T-cell leukemia virus 1 infection, vascular endothelial growth factor (VEGF) signaling pathway, and regulation of actin cytoskeleton (Figure 2(d)).

### 3.5. Crosstalk Genes by Disease-Related Known Genes and DEGs Dysregulated in GEO Datasets

By mapping the periodontitis-related known genes in DisGeNET database to the atherosclerosis-GSE23746 dataset, one group of periodontitis-known genes, including Apolipoprotein L1 (APOL1), C-C Motif Chemokine Ligand 2 (CCL2), and Interferon Stimulated Exonuclease Gene 20 (ISG20), while the other group of periodontitis-known genes, including High Mobility Group Box 1 (HMBG1), CCL5, and MMP8 were downregulated, in the PBMs of atherosclerosis-GSE23746 dataset (Figure 3(a)). Likewise, the expression profiles of atherosclerosis-related known genes in DisGeNET database in the periodontitis-GSE46190 dataset are extracted and displayed in Figure 3(b). A group of atherosclerosis-known genes, such as HMGB1, TNF Superfamily Member (TNFSF) 13B, and IL-18, were upregulated, while another group of atherosclerosis-known genes, such as CD14 Molecule (CD14), Integrin Subunit Beta 2 (ITGB2), and IL1B were downregulated, in the PBMs of periodontitis-GSE46190 dataset (Figure 3(b)).

Figure 3(c) depicts a Venn diagram of 354 crosstalk genes linking atherosclerosis and periodontitis, marked in the shaded emerald color. These 354 crosstalk genes represent the union genes of four categories:

- 165 intersection genes between DEGs dysregulated in atherosclerosis-GSE23746 dataset and DEGs dysregulated in periodontitis-GSE61490 dataset
- 115 intersection genes between atherosclerosis-known genes in DisGeNET and periodontitis-related known genes in DisGeNET
- 28 intersection genes between DEGs dysregulated in atherosclerosis-GSE23746 dataset and periodontitis-related known genes in DisGeNET
- 83 intersection genes between DEGs dysregulated in periodontitis-GSE61490 dataset and atherosclerosis-related known genes in DisGeNET

These 354 genes were defined as the crosstalk genes linking both atherosclerosis and periodontitis and thus were used for the subsequent analysis. Furthermore, Figure 3(c) shows that one gene (HMBG1) was not only a DEG dysregulated in both periodontitis-GSE46190 dataset and atherosclerosis-GSE23746 dataset but also an atherosclerosis- and periodontitis-related known gene in DisGeNET database.

### 3.6. Network Construction

The WGCNA construction processes for atherosclerosis-GSE23746 dataset and periodontitis-GSE61490 dataset are displayed in Figures 4 and 5, respectively. Figures 4(a) and 5(a) show powers for finding a network with scale-free topology properties, of which *β* = 9 (Figure 4(a)) and *β* = 12 (Figure 5(a)) were identified for obtaining scale-free topology by the fit index greater than 0.8. The adjacency matrix was produced through the adjacency function using the identified *β* value and gene expression matrix.  Figure 4(b) shows a plot identifying scale free topology in expression data when the *β* was selected to be 9. In this Log-log plot, the distribution approximately follows a straight line, indicating an approximately scale-free topology. Similarly, Figure 5(b) shows scale free topology in expression data when the *β* was selected to be 12. Figures 4(c) and 5(c) show the gene significance across modules (*p* = 3.4*e* − 19 and *p* = 9.4*e* − 24). Six coexpression modules of each dataset were constructed with various colors (e.g., blue, brown, green, grey, turquoise, and yellow), and the gene number of each module is listed in Table 2. Among the six modules identified in atherosclerosis-GSE23746 dataset, the green and brown modules were found to be with the highest gene significance (Figure 4(c)). Among the six modules identified in periodontitis-GSE61490 dataset, the green module was found to show the highest gene significance (Figure 5(c)). Figures 4(d) and 5(d) show the clustering dendrograms based on the topological overlap together with the assigned module colors. Figures 4(e) and 5(e) show the network heat map plot of (interconnectivity plot) of a gene network together with the hierarchical clustering dendrograms and the six coexpression modules, separately. The heat maps show the progressively darker red denotes, indicating high topological overlap and high coexpression interconnectedness. Figures 4(f) and 5(f) used the scatter plots to show the gene significance for weight versus module membership in the six coexpression modules, respectively. For the atherosclerosis-GSE23746 dataset, the blue module (*p* = 0.00015), brown module (*p* = 1.2*e* − 08), green module (*p* = 0.018), and grey module (*p* = 2.7*e* − 106) exhibited the significant correlation (*p* < 0.05), indicating that hub genes of these modules tend to be highly correlated with weight (Figure 4(f)). For the periodontitis-GSE61490 dataset, the blue module (*p* = 4*e* − 20), brown module (*p* = 1.8*e* − 07), green module (*p* = 2.5*e* − 09), turquoise module (*p* = 7*e* − 14), and yellow module (*p* = 1.4*e* − 07) exhibited significant correlation (*p* < 0.05), indicating that hub genes of these modules tend to be highly correlated with weight (Figure 5(f)).

### 3.7. Identification of Significant Modules

The module eigengene adjacency heat map indicated correlations between any of two modules belonging to the periodontitis-GSE61490 dataset and atherosclerosis-GSE23746 dataset, respectively (Figure 6). As the grey module was unassigned, the turquoise module in the periodontitis-GSE61490 dataset was identified to have the strongest correlation with the turquoise module in the atherosclerosis-GSE23746 dataset (*p* = 3.4*e* − 17) (Figure 6), with the greatest number of the overlapping crosstalk genes (37 crosstalk genes) (Table 3). The second strongest correlation existed between the turquoise module in the periodontitis-GSE61490 dataset and the blue module in the atherosclerosis-GSE23746 dataset (*p* = 1.1*e* − 11) (Figure 6), with 17 overlapping crosstalk genes (Table 3). The third strongest correlation existed between the turquoise module in the periodontitis-GSE61490 dataset and the green module in the atherosclerosis-GSE23746 dataset (*p* = 1.9*e* − 06) (Figure 6), with 4 overlapping crosstalk genes (Table 3). Based on the above correlation values, the turquoise module was selected as the one significant module in the periodontitis-GSE61490 dataset, while blue, green, and turquoise modules were selected as significant modules in the athersclerosis-GSE23746 dataset.

### 3.8. Biological Functions of Crosstalk Genes in the Significant Modules

After extracting the expression profile of crosstalk genes in the significant turquoise module identified in the periodontitis-GSE61490 dataset (Figure 7(a)), the BPs and KEGG signaling pathways enriched by these crosstalk genes were identified (shown in Figures 7(b) and 7(c), respectively). Figure 7(b) shows that organelle-related BPs (e.g., membrane-bounded organelle, intracellular organelle, and intracellular membrane-bounded organelle), metabolic process-related BPs (e.g., organic substance metabolic process, cellular metabolic process, and primary metabolic process) were mainly enriched in this module. Figure 7(c) shows that Ras, calcium, focal adhesion, FoxO, MAPK, oxidative phosphorylation, and metabolic pathways were mainly enriched in this module.

In addition, the expression profiles of crosstalk genes in the three significant modules (turquoise, blue, and green) identified in the atherosclerosis-GSE23746 dataset are displayed in Figures 8(a), 9(a), and 10(a), respectively. The organelle-related BPs (e.g., membrane-bounded organelle, intracellular organelle, intracellular membrane-bounded organelle, organelle lumen, and intracellular organelle lumen) were enriched in all three modules (Figures 8(b), 9(b), and 10(b)), while metabolic process-related BPs (e.g., organic substance metabolic process, cellular metabolic process, and primary metabolic process) were mainly enriched in the turquoise (Figure 8(b)) and blue module (Figure 9(b)). As to the KEGG signaling pathways, platelet activation, insulin, p53, bacterial invasion of epithelial cells, and oxidative phosphorylation pathways were mainly enriched in the turquoise module (Figure 8(c)). The MAPK, AMP-activated protein kinase (AMPK), leukocyte transendothelial migration, phosphatidylinositol 3′-kinase- (PI3K-) Akt, insulin, and platelet activation pathways were mainly enriched in the blue module (Figure 9(c)). Meanwhile, transport, metabolism, absorption, and biosynthesis-related signaling pathways (e.g., synaptic vesicle cycle, mineral absorption, amino sugar and nucleotide sugar metabolism, SNARE interactions in vesicular transport, terpenoid backbone biosynthesis, endocytosis, and glycosaminoglycan biosynthesis-chondroitin sulfate/dermatan sulfate) were mainly enriched in the green module (Figure 10(c)).

### 3.9. Identification of the Core Crosstalk Genes in the Significant Modules

The crosstalk gene-related gene interaction networks for the four significant modules are depicted in Figure 11, and the core crosstalk genes were thus identified. Considering the three significant modules of the atherosclerosis-GSE23746 dataset, two core crosstalk genes Formin Homology 2 Domain Containing 1 (FHOD1) and RAS Guanyl Releasing Protein 2 (RASGRP2) were identified in the blue module (Figure 11(a)), as well as four core crosstalk genes VAMP7, Sorting Nexin 3 (SNX3), Cell Cycle Progression 1 (CCPG1), and PEST Proteolytic Signal Containing Nuclear Protein (PCNP) were identified in the green module (Figure 11(b)), while two core crosstalk genes (HMGB1 and SUMO1) were identified in the turquoise module. Besides, 18 core crosstalk genes were identified in the turquoise module of the periodontitis-GSE61490 dataset (Figure 11(d)), including ATPase H+ Transporting V0 Subunit D1 (ATP6V0D1), Split Hand/Foot Malformation (Ectrodactyly) Type 1 (SHFM1/SEM1), Ubiquinol-Cytochrome C Reductase Core Protein 1 (UQCRC1), Chromosome 14 Open Reading Frame 166 (C14orf166), C9orf78, LSM3 Homolog, U6 Small Nuclear RNA And MRNA Degradation Associated (LSM3), G Protein Subunit Gamma 5 (GNG5), SEC61 Translocon Subunit Gamma (SEC61G), Eukaryotic Translation Initiation Factor 5A (EIF5A), Proteasome 20S Subunit Beta 2 (PSMB2), IMP U3 Small Nucleolar Ribonucleoprotein 3 (IMP3), Catenin Beta Like 1 (CTNNBL1), Selectin P Ligand (SELPLG), FGF1 Intracellular Binding Protein (FIBP), R3H Domain And Coiled-Coil Containing 1 (R3HCC1), N-Acetylneuraminate Synthase (NANS), SYF2 Pre-MRNA Splicing Factor (SYF2), and Eukaryotic Translation Initiation Factor 2 Subunit Beta (EIF2S2).

## 4. Discussion

This study integrated transcriptomes from periodontitis and atherosclerosis and derived crosstalk genes, modules, and enriched biological processes and pathways relevant to periodontitis-atherosclerosis linkage, thereby highlighting key molecular mechanisms that putatively link these two diseases. The core crosstalk genes identified in four significant modules (e.g., RASGRP2, VAMP7, SNX3, HMGB1, SUMO1, FIBP, PSMB2, SELPLG, and SEC61G) were discussed by describing their plausible mechanisms in linking the two diseases.

RASGRP2, a core crosstalk gene identified in the blue module of the atherosclerosis-GSE23746 dataset, is a blood vessel-related gene that can activate platelets by modulating the affinity and avidity of integrins and contribute to the formation of thrombi [29]. Thrombi formation involves procoagulant and proinflammatory serine proteases that lead to the atherosclerotic process by influencing the expression of cytokines and chemokines [30], and RASGRP2 might play a significant role in the initiating atherosclerosis. In addition, RASGRP2 can activate Ras-proximate-1/Ras-related protein 1 (RAP1) and further the proinflammatory process by increasing the production of proinflammatory cytokines, particularly IL-6 and affecting the Nuclear Factor-Kappa B (NF-ĸB) pathway [31]. By promoting thrombi and inflammation, RASGRP2 might play a significant role in the pathogenesis of periodontitis-triggered systemic inflammation-initiated atherosclerosis.

Of the four core crosstalk genes identified in the green module of the atherosclerosis-GSE23746 dataset, VAMP7 is related to another member of VAMP gene family-VAMP3 identified in a GWAS study as a shared susceptibility gene between periodontitis and atherosclerosis. VAMP7 links exocytosis and actin reorganization and thus playing a critical role in platelet activation and platelet granule release [32]. Platelet activation leads to the release of mediators, such as platelet endothelial cell adhesion molecule 1 (PECAM1), RANTES (also known as CCL5), and C-X-C motif chemokine 5 (CXCL5 or ENA78) within platelet granules, promoting cell adhesion, coagulation, proteolysis, and enhanced synthesis of cytokines and chemokines, all of which accelerate the formation of atherosclerotic plaque [33]. VAMP7 has also implicated in regulating inflammation. VAMP7 was able to promote the secretion of proinflammatory cytokine IL12 in dendritic cells [34] and also demonstrated as required for optimal macrophage phagocytosis [35], where TNFɑ plays a central regulating role [36]. Another crosstalk gene-SNX3 is reported as a retromer of promoting Signal Transducer And Activator Of Transcription 3 (STAT3) in cardiovascular diseases [37]. In addition, SNX3 has been suggested as a retromer for Wnt secretion and Wntless (Wls) trafficking [38] in atherosclerosis [39]. Considering the functions of STAT3 [40], Wnt, and Wls signaling in inflammatory bone loss of periodontitis [41, 42], SNX3 can be speculated as an essential regulator in periodontitis, despite no direct experimental evidence.

Two core crosstalk genes, HMGB1 and SUMO1, were identified in the turquoise module of the atherosclerosis-GSE23746 dataset. Substantial evidence supports HMGB1 as a potential therapeutic target in both periodontitis and atherosclerosis, owing to its interaction with Pattern Recognition Receptors (PRR), such as Receptor of Advanced Glycation End-Products (RAGE) and Toll-Like Receptors (TLRs), as well as its activation of inflammatory cytokines IL1B, IL-6, and TNFɑ [43–45]. HGMB1 was found to be upregulated upon periodontal infection, while anti-HMGB1 antibody could suppress the progression of periodontitis through inhibition of inflammatory cytokines, indicating the vital role of HGMB1 in the initiation and progression of periodontitis [46, 47]. In addition, HGMB1 was found to activate peripheral immunity and trigger inflammation in atherosclerosis progression after stroke through binding RAGE and inducing cytokine production in immune cells (monocytes and lymphocytes) [48, 49]. SUMO1, a member of SUMO, is characterized by dynamic and reversible SUMOylation (SUMO conjugation) [50] in multiple cellular activities through modifying posttranslational proteins. SUMO1 is suggested to inhibit NF-ĸB signaling through modification of IĸBɑ (Inhibitor of ĸB) in atherosclerosis [51]. Also, SUMO1 was able to inhibit prolyl-isomerase-1 (Pin1) [52], and downregulation of Pin1 could play a protective role in atherosclerosis [53]. An anti-inflammatory effect of PIN1 inhibition was observed in the periodontal ligament cells induced by nicotine and LPS via blockade of NF-ĸB signaling, implicating Pin1 in periodontitis [51, 54]. SUMO1 may thus regulate the periodontitis-atherosclerosis linkage through Pin1 and NF-ĸB modification [51].

The turquoise module of the periodontitis-GSE61490 dataset identified the greatest number (18) of core crosstalk genes as compared with the other three significant modules. Among these 18 core crosstalk genes, four genes (FIBP, PSMB2, SELPLG, and SEC61G) are supported by experimental evidence. FIBP encodes an intracellular protein that binds selectively to Acidic Fibroblast Growth Factor (aFGF, also named as FGF1), a cytokine that can regulate the inflammatory response [55]. FGF1 was found to promote the phenotypic transition of vascular smooth muscle cells from a contractile phenotype to a secretory phenotype, further resulting in increased expression of proinflammatory chemokines (CXCL9, CXCL10, and CXCL11) [56]. These overproduced chemokines play significant roles in facilitating leukocyte infiltration and atherosclerotic plaque formation [56]. Evidence related to FGF1 effects on inflammatory response in periodontitis is not available to our knowledge. However, another member of the FGF family-FGF2 can inhibit periodontal inflammation by inhibiting CD40 signaling and decreasing the expression of proinflammatory cytokines (IL6 and TNFɑ) [57]. PSMB2 plays a critical role in releasing peptides by regulating the ubiquitin-proteasome pathway in various cellular processes [41]. The Ubiquitin–Proteasome System (UPS) can activate NF-ĸB [41], which is a master regulator of inflammatory and immune responses through regulation of cytokines (ILl, IL6, and TNFɑ) and cell adhesion molecules (Intercellular Adhesion Molecule (ICAM) 1, Vascular Cell Adhesion Molecule (VCAM) 1, E-selectin) in periodontitis and atherosclerosis [42, 58]. In addition, proteasome downregulation has the potential to attenuate atherosclerotic inflammation, further resulting in plaque destabilization [58]. Thus, the involvement of PSMB2 in the periodontitis-atherosclerosis linkage seems plausible. In case of SELPLG, the several studies have focused on its role mediating the pathogenesis of atherosclerosis. SELPLG was found to promote the development of atherosclerosis via mechanisms of regulating glucose metabolism, lipid metabolism, amino acid, and phospholipid metabolism, activating and recruiting leukocytes, and promoting the adhesive interactions between endothelial cells and leukocytes [59, 60]. Another study showed that SELPLG could significantly promote systemic inflammatory responses by upregulating the expression levels of proinflammatory cytokines (TNFɑ and IL6) [61]. However, whether periodontitis-triggered systemic inflammation can lead to the upregulation of SELPLG has not been investigated. Considering SEC61G, the Sec61 complex has been demonstrated to be the central component of the protein translocation apparatus of the endoplasmic reticulum (ER) membrane [62]. Increasing evidence shows that the ER stress signaling pathway is involved in pathological conditions including periodontitis and atherosclerosis. ER signaling reportedly contributes to the progression of periodontitis by two ways: the induction of apoptosis and upregulating inflammatory response by activating the proinflammatory NF-ĸB pathway [63]. ER stress is implicated in the pathogenesis of atherosclerosis, and prolonged ER stress is a significant contributing factor in the proatherogenic progression of the atherosclerotic lesions by inducing apoptosis of lesional macrophages and enhancing oxidative stress-mediated damage of vascular cells [64].

In line with previous studies, several inflammatory and immune signaling pathways, such as the bacterial invasion of epithelial cells, platelet activation, and MAPK signaling pathway, were found primarily enriched by the crosstalk genes in the significant modules. Bacterial invasion of epithelial cells could be an essential link between periodontitis and atherosclerosis, as periodontal pathogen burden may be contributed to atherosclerosis progression [1]. Additionally, platelet activation might link atherosclerosis with periodontitis [65]. The platelets activated by periodontal pathogen burden can further promote the production of proinflammatory cytokines, thus accentuating risk for atherosclerosis and increased platelet activation induced procoagulant, and inflammatory state in periodontitis is recognized [65–68]. Furthermore, MAPK signaling has been implicated in atherosclerosis and periodontitis, given its role in promoting inflammatory responses. The activation of MAPK signaling axis was shown to contribute to the severity of periodontitis by promoting bone destruction and periodontal inflammation via upregulating IL1*β*, IL6, TNFɑ, MMP13, and Receptor Activator of Nuclear Factor Kappa-B Ligand (RANKL) [69]. The LPS-activated MAPK was shown to be a key driver of atherosclerosis by playing proapoptotic, proinflammatory, and antiproliferative roles via activating its downstream targets-MAPK-Activated Protein Kinase 2 (MAPKAPK2/MK2) and the Heat Shock Protein 27 (HSP27) [70]. Of note, some biological processes, such as cellular response to reactive oxygen species and increased oxygen levels, were identified in the enrichment analysis, indicating oxidative stress as a shared pathology in periodontitis and atherosclerosis [71].

It is important to highlight why PBMs were selected for investigation in the current research. The innate immune effector role of PBMs in the pathogenesis of both diseases is one reason for our focus. Another reason is that the gene expression is typically tissue-specific; thus, a disease may cause a certain gene to be upregulated in one tissue but downregulated in another type of tissue. Thus, comparing the genetic alterations of distinct tissue (gingival tissue, atherosclerotic plaques) may be less biologically meaningful. The gene expression alterations in PBMs in periodontitis and atherosclerosis were therefore selected for analysis in the current study.

This study bears some potential limitations. The present work included the publicly available microarray/RNA-sequencing data for periodontitis vs. control and atherosclerosis vs. control cases that originated from different populations. The lack of data from patients with both periodontitis and atherosclerosis is the greatest limitation of this study, and the future research should validate these findings in cohorts with both diseases. Within the limitations of this study, the genetic crosstalk markers identified can be considered as the preliminary basis for new hypotheses which can direct targeted experimentation and validation in future research.

Taken together, the most important finding in our study was the identification of putative significant crosstalk genes involved in shared molecular mechanisms between atherosclerosis and periodontitis. Although the experimental validation of these purported linkage genes was not performed, these findings were broadly supported by existing experimental evidence. Therefore, these findings from mining experimental transcriptomes could be considered as well-supported hypotheses, for directing research in the context of pathophysiology of CP-atherosclerosis linkage. Simultaneously, these data also provide new directions for future translational research for drug development and risk mitigation for both diseases.

## 5. Conclusion

Exploration of available transcriptomic datasets revealed crosstalk genes (e.g., RASGRP2, VAMP7, SNX3, HMGB1, SUMO1, FIBP, PSMB2, SELPLG, and SEC61G) and significant pathways (bacterial invasion of epithelial cells, platelet activation, and VEGF signaling pathway) as the top candidate molecular linkage mechanisms between atherosclerosis and periodontitis.

## Figures and Tables

**Figure 1:** Work flowchart.

**Figure 2:** Identification of the overlapping DEGs shared between periodontitis-GSE46190 dataset and atherosclerosis-GSE23746 dataset. (a) The Venn diagram showing the overlapping 165 DEGs dysregulated in both periodontitis-GSE61490 and atherosclerosis-GSE23746 datasets. (b) The protein-protein interaction (PPI) network that was constructed based on the 165 overlapping DEGs dysregulated in both periodontitis and atherosclerosis. (c) The biological processes that were significantly enriched by the overlapping 165 DEGs. (d) The signaling pathways that were significantly enriched by the overlapping 165 DEGs.

**Figure 3:** Identification of crosstalk genes linking atherosclerosis and periodontitis. (a) Heat map showing the expression pattern of DisGeNET-periodontitis-related known genes mapped to the atherosclerosis-GSE23746 dataset. (b) Heat map showing the expression pattern of the DisGeNET-atherosclerosis-related known genes mapped to the periodontitis-GSE46190 dataset. (c) Venn diagram to identify crosstalk genes linking atherosclerosis and periodontitis, via intersecting any two groups of genes belonging to the four groups (i.e., DEGs dysregulated in atherosclerosis-GSE23746 dataset, DEGs dysregulated in periodontitis-GSE61490 dataset, atherosclerosis-related known genes in DisGeNET, and periodontitis-related known genes in DisGeNET). The 354 crosstalk genes identified by the Venn diagram were displayed in the shared emerald color.

**Figure 4:** Identification of significant modules in atherosclerosis-GSE23746 dataset by performing WCGNA analysis. (a) Scale-free fit index for different powers (*β*) and mean connectivity analysis for various soft threshold powers (*β*). (b) Log-log plot of the whole-network connectivity distribution showing the quality of relationship between connectivity (*k*) and *P*(*K*), when power *β* was selected to be 9. *X*-axis: the logarithm of whole network connectivity; *Y*-axis: the logarithm of the corresponding frequency distribution. (c) Bar plot of mean gene significance (*p* = 3.4*e* − 19) across six coexpression modules constructed with various colors (e.g., blue, brown, green, grey, turquoise, and yellow). The higher the mean gene significance in a module, the more significantly related the module is to the clinical trait of interest. (d) Gene dendrogram obtained by average linkage hierarchical clustering. The color row underneath the dendrogram shows the module assignment determined by the Dynamic Tree Cut. (e) Network heat map plot of topological overlap in the gene network. In the heat map, each row and column correspond to a gene, light color denotes low topological overlap, and progressively darker red denotes higher topological overlap. Darker squares along the diagonal correspond to modules. The gene dendrogram and module assignment are shown along the left and top. (f) The scatter plots of gene significance versus intramodular *k* in the different modules of atherosclerosis-GSE23746 dataset.

**Figure 5:** Identification of interesting modules in the periodontitis-GSE61490 dataset by performing WCGNA analysis. (a) Scale-free ft index for different powers (*β*) and mean connectivity analysis for various soft thresholding powers (*β*). (b) Log-log plot of the whole-network connectivity distribution showing the quality of relationship between connectivity (*k*) and *P*(*K*), when power *β* was selected to be 12. *X*-axis: the logarithm of whole network connectivity; *Y*-axis: the logarithm of the corresponding frequency distribution. (c) Bar plot of mean gene significance (*p* = 9.4*e* − 24) across six coexpression modules constructed with various colors (e.g., blue, brown, green, grey, turquoise, and yellow). The higher the mean gene significance in a module, the more significantly related the module is to the clinical trait of interest. (d) Gene dendrogram obtained by average linkage hierarchical clustering. The color row underneath the dendrogram shows the module assignment determined by the Dynamic Tree Cut. (e) Network heat map plot of topological overlap in the gene network. In the heat map, each row and column correspond to a gene, light color denotes low topological overlap, and progressively darker red denotes higher topological overlap. Darker squares along the diagonal correspond to modules. The gene dendrogram and module assignment are shown along the left and top. (f) The scatter plots of gene significance versus intramodular *k* in the different modules of periodontitis-GSE61490 dataset.

**Figure 6:** The module eigengene adjacency heat map shows the correlations between coexpression modules in GSE61490 and GSE23746 datasets. The horizontal axis represents the six coexpression modules in the atherosclerosis-GSE23746 dataset, and the vertical axis represents the six coexpression modules in the periodontitis-GSE61490 dataset. Colors correspond to correlations, in which darker red color represents high correlation, and lighter red means low correlation. The number of overlapped crosstalk genes and *p* values is also labeled.

**Figure 7:** The expression pattern of genes in the significant turquoise module of periodontitis-GSE61490 dataset. (a) Heat map showing the expression profiles of genes in the turquoise module of periodontitis-GSE61490 dataset. (b) The biological processes significantly enriched by the genes in the turquoise module of periodontitis-GSE61490 dataset. (c) The signaling pathways significantly enriched by the genes in the turquoise module of periodontitis-GSE61490 dataset.

**Figure 8:** The expression pattern of genes in the significant turquoise module of atherosclerosis-GSE23746 dataset. (a) Heat map showing the expression profiles of genes in the turquoise module of atherosclerosis-GSE23746 dataset. (b) The biological processes significantly enriched by the genes in the turquoise module of periodontitis-GSE23746 dataset. (c) The signaling pathways significantly enriched by the genes in the turquoise module of atherosclerosis-GSE23746 dataset.

**Figure 9:** The expression pattern of genes in the significant blue module of atherosclerosis-GSE23746 dataset. (a) Heat map showing the expression profiles of genes in the blue module of atherosclerosis-GSE23746 dataset. (b) The biological processes significantly enriched by the genes in the blue module of periodontitis-GSE23746 dataset. (c) The signaling pathways significantly enriched by the genes in the blue module of atherosclerosis-GSE23746 dataset.

**Figure 10:** The expression pattern of genes in the interested green module of atherosclerosis-GSE23746 dataset. (a) Heat map showing the expression profiles of genes in the green module of atherosclerosis-GSE23746 dataset. (b) The biological processes significantly enriched by the genes in the green module of periodontitis-GSE23746 dataset. (c) The signaling pathways significantly enriched by the genes in the green module of atherosclerosis-GSE23746 dataset.

**Figure 11:** The crosstalk gene-related gene interaction networks of the four significant modules: (a) crosstalk gene-related network of the green module in the atherosclerosis-GSE23746 dataset; (b) crosstalk gene-related network of the turquoise module in the atherosclerosis-GSE23746 dataset; (c) crosstalk gene-related network of the turquoise module in the atherosclerosis-GSE23746 dataset; (d) crosstalk gene-related network of the turquoise module in the periodontitis-GSE41690 dataset. Round nodes with yellow color: crosstalk genes dysregulated in the atherosclerosis-GSE23746 dataset; round nodes with rose red color: crosstalk genes dysregulated in the periodontitis-GSE61490 dataset; diamond nodes with the rose red border: crosstalk genes dysregulted in both atherosclerosis-GSE23746 dataset and periodontitis-GSE61490 dataset; round nodes with the sky blue color: noncrosstalk genes which interact with the crosstalk genes.

**Table 1:** The topological characteristics of the top 30 nodes with the greatest degree in the 165 overlapping DEG-based PPI network shown in Figure 2(b), ranked in the descending order of degree.

Name	Degree	Average shortest path length	Betweenness centrality	Closeness centrality	Clustering coefficient	Topological coefficient
APP	2209	2.0703	0.5313	0.4830	0.0002	0.0011
SUMO1	802	2.3347	0.1769	0.4283	0.0009	0.0021
GABARAPL1	534	2.6731	0.0912	0.3741	0.0013	0.0043
SRC	488	2.7686	0.0958	0.3612	0.0005	0.0057
CSNK2B	294	2.7594	0.0525	0.3624	0.0016	0.0063
OFD1	258	2.8469	0.0482	0.3513	0.0016	0.0074
CDK4	215	2.5037	0.0339	0.3994	0.0049	0.0059
AP2M1	214	2.8266	0.0328	0.3538	0.0036	0.0089
TUBA1C	192	2.7066	0.0236	0.3695	0.0081	0.0088
NUDC	160	2.8917	0.0286	0.3458	0.0017	0.0120
ACTN1	150	2.6568	0.0242	0.3764	0.0094	0.0097
RPL17	150	2.8182	0.0129	0.3548	0.0056	0.0110
SHFM1	137	2.9457	0.0170	0.3395	0.0013	0.0224
ITGB1	134	2.9170	0.0188	0.3428	0.0028	0.0158
U2AF1	131	2.9573	0.0120	0.3381	0.0000	0.0321
UBC	129	2.0214	0.1225	0.4947	0.0109	0.0139
PDLIM7	128	2.8821	0.0179	0.3470	0.0066	0.0144
TAGLN2	127	2.5288	0.0183	0.3954	0.0126	0.0099
NR4A1	125	2.8661	0.0173	0.3489	0.0028	0.0120
PSMB5	119	2.8568	0.0100	0.3500	0.0182	0.0152
HMGB1	114	2.9565	0.0152	0.3382	0.0000	0.0287
FKBP8	100	2.9373	0.0091	0.3404	0.0160	0.0235
SSBP1	99	2.8495	0.0104	0.3509	0.0099	0.0160
PSMB2	97	2.8640	0.0078	0.3492	0.0253	0.0168
SNX3	91	2.8637	0.0109	0.3492	0.0085	0.0160
PTPN12	82	2.6034	0.0141	0.3841	0.0057	0.0133
UNC45A	82	2.9257	0.0076	0.3418	0.0066	0.0226
TPM4	79	2.9301	0.0068	0.3413	0.0110	0.0252
NMI	79	2.9721	0.0125	0.3365	0.0003	0.0204
EIF2S2	77	2.5806	0.0110	0.3875	0.0116	0.0152

**Table 2:** The number of crosstalk genes in different coexpression modules of periodontitis-GSE61490 dataset and atherosclerosis-GSE3746 dataset.

Coexpression modules	Number of genes in the periodontitis-GSE61490 dataset	Number of genes in the atherosclerosis-GSE23746 dataset
Blue	56	293
Brown	49	47
Green	20	30
Grey	366	1749
Turquoise	665	471
Yellow	21	31

**Table 3:** The correlations between significant modules.

GSE61490	GSE23746	Fisher (*p* value)	Overlapping crosstalk genes (number)
Turquoise	Turquoise	3.4*e*-17	37
Turquoise	Blue	1.1*e*-11	17
Turquoise	Green	1.9*e*-06	4

## Data Availability

The datasets used and/or analyzed during the current study are available from the corresponding author on reasonable request.
